# Analysis of the Outcome of Treatment of Brain Metastases from Malignant Trophoblastic Tumours and Risk Factors for Prognosis during Pregnancy

**DOI:** 10.1155/2022/3932460

**Published:** 2022-08-11

**Authors:** Anbang Wang, Hua Zhang

**Affiliations:** ^1^Department of Neurosurgery, The First People's Hospital of Xianyang, Xianyang 712000, Shaanxi, China; ^2^Department of Gynaecology and Obstetrics, The Second Affiliated Hospital of Shaanxi University of Chinese Medicine, Xianyang 712000, Shaanxi, China

## Abstract

Temozolomide combined with whole-brain radiotherapy has good near-term efficacy and safety in the treatment of brain metastases from nonsmall cell lung cancer. In this study, we analyzed the risk factors for treatment and prognosis of brain metastases in gestational trophoblastic neoplasm (GTN) during pregnancy. Thirty-one patients with brain metastases were included in the study. All patients had a pathological diagnosis of primary lesions, including 23 adenocarcinomas, 7 squamous carcinomas, and 1 adenosquamous carcinoma, and had ≥3 intracranial metastases, controlled primary lesions (including resected primary lesions or unresectable primary lesions in partial remission (PR)/complete remission (CR) for ≥2 months) by cranial enhancement MRI and no extracranial metastases. Presence or control of extracranial metastases was for ≥2 months. The common adverse toxic effects were nausea, vomiting, neutropenia, and thrombocytopenia, but most patients tolerated them with symptomatic management.

## 1. Introduction

Gestational trophoblastic neoplasm (GTN) is the only gynecologic malignancy associated with pregnancy that can be cured by chemotherapy. To date, the incidence of GTN has not been clearly documented and varies widely between different regions of the world [1–4], with approximately 1 case per 300–500 pregnancies in Southeast Asian countries. According to the FIGO (International Federation of Obstetricians and Gynecologists)/WHO outcome scoring system (2000), GTN is classified into low-risk (≤6) and high-risk (≥7) systems. The 2018 FIGO cancer report [5] and the 2013 ESMO clinical practice guidelines [6] recommend monotherapy for low-risk patients and recommend either the actinomycin D (ACTD) or methotrexate (MTX) regimens for monotherapy. Although GTN is very sensitive to chemotherapy, some patients still develop resistance. Studies have shown [7] that low-risk patients are 9–33% more likely to switch to combination regimens due to drug resistance or side effects. In recent years, with the advancement of basic research, immunotherapy and targeted therapy have become two hot spots in oncology treatment. To improve the efficacy of brain metastases, the use of chemotherapy and molecularly targeted drugs has received increasing attention in recent years, but the efficacy of many chemotherapy regimens is unsatisfactory because most chemotherapeutic agents cannot cross the blood-brain barrier and have severe neurotoxic adverse effects. Standard targeted therapy is for EGFR-mutant NSCLC. For example, for standard targeted therapy in EGFR-mutant NSCLC, both gefitinib and erlotinib are suboptimal, which is associated with poor intracranial control [8].

Basic research [9] and targeted therapies [10] in GTN immunotherapy have made great progress and have shown initial success in the clinical management of drug-resistant or refractory GTN. In this article, we review the progress of clinical research on immunotherapy and targeted therapy for GTN with the aim of providing clinical support for the treatment of drug-resistant and refractory GTN.

## 2. Immunotherapy

### 2.1. Immunotherapy Targets

GTN is as immunogenic as normal gestational trophoblast cells and stimulates an immune response from the maternal immune system, but GTN successfully evades immune surveillance and modulates the maternal placental and peripheral immune systems and then rapidly proliferates, grows, invades, and metastasises widely. Drug resistance or refractory to treatment is the main reason for the failure of GTN treatment, and therefore, immunotherapy is becoming a hot topic for exploratory research in this area [11].

By analyzing the expression of PD-L1 in the tumor tissues of GTN patients, all choriocarcinoma tissues (*n* = 63), epithelial GTN tissues (*n* = 12), and placental GTN tissues (*n* = 41) were found to be positive for PD-L1, most of which were strongly positive [12]. It was also confirmed that PD-L1 was positively expressed in all GTN tissues and that its expression was not associated with FIGO score or prechemotherapy outcome [13],suggesting that PD-L1 plays a key role in the development and progression of GTN [14].

### 2.2. Immune Checkpoint Inhibitors

PD-L1 blocking monoclonal antibodies, such as the anti-PD-1 drug pembrolizumab, have shown promising clinical results in a variety of malignancies. Studies have shown that immune checkpoint inhibitors can significantly improve the outcomes of patients with GTN, especially those with drug-resistant or refractory GTN. In 2017, a case of very high-risk (stage IVB, FIGO prognosis score of 18) GTN treated with pabolizumab was reported to have a favourable outcome [15]. The patient was a 26-year-old woman with liver metastases at clinical diagnosis and was treated with 2 courses of EP (etoposide + cisplatin) induction chemotherapy and 4 courses of EMACO (etoposide + methotrexate + actinomycin D/cyclophosphamide + vincristine), with a fall and then a rise in blood HCG.

The patient was treated with pabolizumab 200 mg (21 d in 1 cycle). At the time of writing, 3 courses of treatment had been administered and the symptoms associated with brain metastases had resolved significantly, and HCG had decreased to normal levels. After 2 courses of pabolizumab treatment, hepatic impairment of degree III was observed, but liver function returned to normal with hepatoprotective therapy and did not affect subsequent treatment. No other grade III-IV drug toxicities were observed during pabolizumab treatment. Four patients with GTN at very high risk of liver or brain metastases were reported to be treated with pabolizumab. All patients were treated with pabolizumab 2 mg/kg for 21 d for 5 courses, resulting in complete remission in 3 patients and death due to progression in 1 patient [16]. Two cases of very high-risk GTN treated with pabolizumab were reported with equally satisfactory results [17]. In this study, one patient treated with pabolizumab 200 mg (21 d course) was assessed to be in complete remission on imaging after 5 courses and entered clinical follow-up; the other patient had been treated for 3 courses at the time of writing and was also in complete remission, with no grade III-IV side effects. In summary, although the clinical studies of immunotherapy in GTN are few and small and the level of clinical evidence is low, the exploratory studies in very high-risk patients and relapsed drug-resistant refractory patients have achieved encouraging results and have helped in the clinical management of these patients.

## 3. Targeted Therapy

With the advancement of molecular typing of malignant tumours and hereditary tumours and the rapid development of biologically targeted therapies, the treatment of malignant tumours has gradually entered the era of precision medicine. In recent years, the clinical application of targeted therapies in GTN has also made breakthroughs.

### 3.1. VEGF Targeted Therapy

The expression of VEGF in GTN tissues was found to be significantly higher in normal placental tissues than in staphyloma tissues, and the expression of VEGF, angiopoietin-1, and angiopoietin-2 was also significantly higher in placental GTN tissues than in choriocarcinoma tissues [18]. Antiangiogenic therapy increases endothelial glycoprotein expression, and blockade of endothelial glycoproteins increases VEGF expression. Although the expression of endothelial glycoprotein is limited outside the endothelium, it is a very specific marker of placental syncytial trophoblast cells and an ideal histopathological marker in choriocarcinoma tissue. This scholar reported a satisfactory clinical outcome in a patient with refractory choriocarcinoma treated with bevacizumab [19]. The patient was a 36-year-old female with low-risk GTN at the time of presentation. The patient's HCG decreased to normal after 4 courses of treatment. The patient was assessed to be in complete remission after 4 courses of treatment, and at the time of writing, the patient had been followed up for 28 months. Unfortunately, the study did not report in detail the treatment interval and the specific use of TRC105 or the drug-related side effects of bevacizumab.

### 3.2. EGFR Targeted Therapy

The epithelial growth factor receptor (EGFR) is a transmembrane glycoprotein located on the surface of the cell membrane and is a member of the ErbB family of conserved receptors. EGFR acts by influencing tumour cell proliferation, invasion, metastasis, and apoptosis. In vitro studies found that EGFR and HER2 were significantly overexpressed in GTN cells and that lapatinib significantly inhibited tumour cell growth by regulating the expression of EGFR and HER2 in GTN. To investigate the expression pattern of c-ErbB2 and Bcl-2 proteins in staphylococcal tissues, they performed immunohistochemical analysis on 220 pregnancies, including 39 aborted tissues and 41 partial and 140 complete staphylococcal tissues [20]. The results showed that c-ErbB2 expression was observed in 3 partial and 10 complete gravida and that Bcl-2 immunostaining was more pronounced in partial (61%) and complete gravida (70.7%) than in aborted tissues. In conclusion, EGFR-related targets may become new targets for the treatment of GTN, but there is a lack of clinical studies on EGFR in GTN, and further research is needed to determine whether its related drugs have clinical application.

### 3.3. Through-Targeted Therapy

Current research in GTN targeting also includes targeting abnormal pathways, such as the PI3K/AKT pathway. Activation of the PI3K/AKT signaling pathway was found to stimulate the proliferation of GTN cells, while lapatinib inhibited the proliferation of GTN cells by blocking the PI3K/AKT signaling pathway [21]. The mechanism by which apigenin inhibited the growth of choriocarcinoma cells was investigated, and apigenin was found to decrease the viability and mobility of JAR and JEG3 cells, increase apoptosis, and inhibit mitochondrial membrane potential [22]. Gene sequence analysis of uterine cavity tissues from eight GTN patients confirmed that PTEN and PI3K-AKT signaling pathways could be optional targets for clinical treatment of GTN [23].

## 4. Materials and Methods

### 4.1. Clinical Information

The incidence of brain metastases was 0.36% in 3 cases and renal metastases was 0.12% in 1 case. The incidence of metastases to the brain was 0.95% in 735 patients with choriocarcinoma and 1.1% in 8 patients with metastases to the kidneys; 2 patients had metastases to both the brain and kidneys, with an incidence of 0.27%. In this group of 19 patients, the age ranged from 22 to 48 years old, with an average of 29.8 years old.

### 4.2. Diagnosis

In 5 cases, the last pregnancy was gravida, in 10 cases, early pregnancy, in 2 cases, full-term delivery, in 1 case, ectopic pregnancy, and in 1 case, rupture of the right uterine horn. 17 of the 19 cases had pulmonary metastases, 8 cases had cerebral metastases, 2 cases had vaginal metastases, and 4 cases had pelvic organ metastases.

All patients underwent blood tests for HCG and 13-IaCC, abdominal ultrasound or CT, pelvic ultrasound, lung CT, or lung X-ray. Some patients underwent cerebroscopy and intravenous pyelogram.

### 4.3. Treatment

Four patients were critically ill at the time of admission and died of respiratory and circulatory failure or hepatic coma after only one course of chemotherapy or without chemotherapy. The remaining 15 patients received a multidrug combination regimen of 2–22 courses of chemotherapy, with an average of 8.9 courses. The main chemotherapy regimens were 5-fluorouracil (5-FU) based multidrug combinations ((5-FU + vincristine (KSM) + vincristine (VCR) or 5-FU + KSbf + abscisicidal mustard (ATl258) + VCR) or the EMACO regimen.

Five patients received 1–5 courses of 5-FU brain perfusion in conjunction with systemic chemotherapy, with an average of 3.4 courses. The average number of sessions was 4. The interval between each session was 2-3 d.

Among the patients who received more than 2 courses of chemotherapy, the 5 patients with brain metastases received subarachnoid puncture intrathecal MTX at 10–15 rag each time, 3-4 times a course. 17 courses of MTX were given intrathecally to the 5 patients, an average of 3.4 courses per patient.

Tube chemotherapy or embolization: in five cases, the uterine artery was cannulated six times for uterine lesions, one case was cannulated for suspected renal metastases, one case was cannulated for hepatic metastases, and one case was embolised with bilateral supracerebral, uterine, and internal iliac arteries for hematuria with bleeding from vaginal metastases.

Twelve of the 19 cases were treated with a total of 15 different procedures. Four cases underwent total hysterectomy with double adnexal resection and high ligation of both ovarian arteries, and one case underwent simultaneous resection of a brain metastasis and brain repair. The remaining five cases were treated surgically at outside hospitals. Two cases underwent dissection, two cases underwent craniotomy, and one case underwent total hysterectomy + right fallopian tube + part of right ovary + part of small intestine + appendix.

### 4.4. Observation Indicators

1. Treatment effect: the clinical treatment effect is evaluated according to the efficacy evaluation criteria of solid tumors, including four criteria: complete remission (CR), partial remission (PR), no change (SD), and progression (PD), and the effective rate is PR and CR.
2. Analysis of influencing factors: gender, number of metastases, RPA classification, MMSE score before radiotherapy, extracranial metastasis, and other factors
3. Analysis of toxicity and adverse reactions: including hematological toxicity, leukopenia, thrombocytopenia, gastrointestinal toxicity, nausea and vomiting, and diarrhea, except for drug-resistant patients, the main manifestation of drug resistance is the enlargement of lesions by more than 50% compared to pretreatment or the appearance of new distant metastases
4. Quality of life assessment: the SF-36 scale was used to evaluate patients' “social, emotional, cognitive, and spiritual functions. The total score of each function was 100 points, and the score was directly proportional to the patients' quality of life.

### 4.5. Statistical Methods

The collected data were entered into the Excel table, and statistical SPSS 22.0 software was used to analyze the data. If the collected data met the normal distribution, composition ratio, and rate description of count data, measurement data were expressed as (mean ± standard difference) and *t*-test. *P* < 0.05 has statistical significance as GraphPad Prism8.

## 5. Results

Of the 19 patients, four were admitted to the hospital and died of liver coma or respiratory and circulatory failure without chemotherapy or after only one course of chemotherapy because they were nearing the end stage of metastasis in multiple organs. Out of the other 15 patients, 11 patients achieved complete remission after 2–22 courses of chemotherapy, 2 patients survived with tumours in their lungs after normalisation of their blood biochemical parameters, and 2 patients were discharged after 7 and 14 courses of chemotherapy, respectively. The complete remission rate was 73.3% (11/15). The 11 patients in complete remission were followed up regularly after discharge, the shortest being 4–43l-months and the longest being 6 years, with no signs of recurrence. Two patients with residual lung tumours survived, one for 8 years and the other for 6 months, with normal blood 13-HCG.

The objective remission (ORR) rate was 74.1% (23/31), with a CR rate of 19.3% (6/31) and a PR rate of 54.8% (17/31) (Figure 1).

The neurological symptoms (headache, nausea, vomiting, memory loss, and cognitive impairment) in 25 of the 31 patients before enrollment were significantly improved in 12 patients and slightly improved in 8 patients after treatment, resulting in a neurological remission rate of 80%. As of 1^st^ August 2016, of the 31 patients, 16 had intracranial progression, 8 had progression of the original lesion, 5 had new lesions, and 3 had progression of the original lesion with new lesions, of which 7 were treated locally with gamma knife, 3 were treated surgically, and the rest were treated symptomatically. Out of the 23 deaths, 5 were due to brain herniation due to intracranial progression and the rest to systemic failure due to combined liver, bone, and other systemic metastases. The median time without intracranial progression was 11.5 months, the median survival time was 13 months, and the 1-year PFS and OS were 63.1% and 64.5%, respectively (Figures 2 and 3).

Univariate analysis showed that the presence of extracranial metastases and preradiotherapy MMSE score were statistically significant for PFS (*P* < 0.05) (Table 1). Sex, number of metastases (>3 vs = 3), RPA grade, and preradiotherapy MMSE score were statistically significant for OS (*P* < 0.05). Multifactorial analysis showed that preradiation MMSE score (27–30 vs <27) was an independent prognostic factor for PFS and RPA grade (grade 1 vs. grade 2) and was an independent prognostic factor for OS (Table 2).

Toxic adverse reactions during the administration of TMZ were mainly hematological and gastrointestinal. No liver, kidney, or cardiac related toxicity was observed in this group and there were no treatment-related deaths (Table 3, Figure 4).

After treatment, the social, emotional, cognitive, and spiritual functions increased significantly in both groups, as shown in Figure 5.

## 6. Discussion

Patients with metastatic brain metastases from choriocarcinoma or erosive staphyloma often have clinical symptoms such as hematuria and difficulty in urination. In combination with ultrasound and other imaging studies, early detection and treatment are often possible.

### 6.1. Treatment of Brain and Kidney Metastases

In our group of 19 patients, apart from 4 brain metastases who died of severe disease, the remaining 15 patients were treated with complete remission in 11 cases, partial remission in 2 cases, and progressive disease in 2 cases. Most of the patients were treated with 5-Fu-based combination chemotherapy (e.g., 5-FU + SM + VCR or 5-FU + KSM + ATl258 + VCR) or EMA/CO regimens. To enhance the efficacy, 5-FU cerebral perfusion can be administered concurrently during or before each course of treatment for brain metastases, with a reduced amount of systemic intravenous dosing. In 5 of the 19 cases in this group, 5-FU brain perfusion was administered in parallel with systemic chemotherapy. 5-FU brain perfusion can maintain a higher concentration of the drug in the brain while keeping the total amount of 5-FU virtually unchanged, resulting in better efficacy and fewer adverse effects. The treatment of renal metastases, once clearly diagnosed in the early years, was usually surgical removal of the affected kidney. Since 5-FU chemotherapy has proved to be effective, chemotherapy alone has been used for those with less severe bleeding. However, if severe bleeding occurs, the kidney is also removed and postoperative chemotherapy is given.

### 6.2. Differences in Prognosis between Brain and Kidney Metastases

In this group, two patients had both renal and brain metastases, of which one was in complete remission and one died. The prognosis of brain metastases was better than that of kidney metastases, which was considered to be related to the following factors. (1) Differences in disease: the prognosis of brain metastases is not uncommon in gestational trophoblastic tumours and the incidence of brain metastases has been reported in the literature to range from 8% to 28% BJ. Once brain metastases occur, the condition is more dangerous and is one of the main causes of death. The prognosis of brain metastases combined with liver metastases is the worst, and none of the 10 cases of brain-hepatic metastases in this study survived ∞ J. Another study reported that the 5-year survival rate of patients with liver-brain metastases was only 10%. In this study, there were no cases of brain metastases combined with liver metastases. (2) Patients with brain metastases who received systemic chemotherapy and 5-FU cerebral perfusion had a significant effect. Four of the patients with brain metastases were cured by 5-FU cerebral perfusion, while one case had combined brain and kidney metastases. The 5-FU cerebral perfusion can maintain a high local concentration of the drug in the brain while keeping the total amount of 5-FU virtually constant [24].

### 6.3. Differences in the Pathways of Brain and Kidney Metastases

The primary focus of malignant trophoblastic tumours usually originates in the uterus and develops outward from the uterus after a certain period of time [21]. After a certain period of time, the tumour cells multiply and grow, penetrating the vessel wall and invading the alveoli, developing into a metastatic tumour. Pulmonary metastases are the most common of all organs [22]. The incidence of pulmonary metastases in combination with renal metastases is higher, which is thought to be related to the fact that renal metastases are secondary to pulmonary metastases. The incidence of kidney metastases in combination with lung metastases is higher and is thought to be related to the secondary development of kidney metastases in the lung. The intrapulmonary metastases invade the pulmonary veins, return to the left heart, and then spread to the kidney via the body circulation. The incidence of brain metastases in combination with pulmonary metastases is also high, suggesting that hematogenous metastases are also a major route of brain metastases. Some patients with brain metastases do not have pulmonary metastases but do have vaginal and pelvic metastases, which are considered to be local infiltrations.

Most chemotherapeutic drugs are only moderately active in brain metastases, with nitrosoureas, temozolomide, topotecan, and leucovorin showing high concentrations in the brain. In breast cancer, small-molecule targeted drugs such as neratinib in combination with capecitabine also showed good ORR for intracranial metastases, and large-molecule monoclonal antibodies such as T-DM1 also showed some efficacy, probably due to heterogeneous leakage of the blood-tumor barrier [23]. In terms of immunotherapy, immunotherapy of brain metastases from lung cancer and melanoma has been studied more frequently and has shown some promising results. For patients with brain metastases from advanced tumors, some regimens can be selected according to NCCN guidelines, CSCO guidelines, and ESMO guidelines.

Research on brain metastases has never stopped, and new compounds with higher molecular specificity, including higher blood-brain barrier and blood-tumor barrier permeability, are being developed. Strategies to increase drug delivery across the blood-brain barrier are also being investigated, including opening the tight junctions of the blood-brain barrier, inhibiting the blood-brain barrier efflux pump system, optimizing drug selection, and optimizing drug delivery [25]. The study also aims to optimize drug selection and drug delivery for better prognosis of patients with brain metastases.

In conclusion, brain metastases from trophoblastic tumours can be treated with whole-body chemotherapy based on 5-FU or EMA/CO regimens, supplemented by local infusion of 5-FU into the brain. The main route of metastasis for renal metastases is blood transfer, whereas brain metastases may be mainly from local infiltration. Patients with renal metastases have a poorer prognosis than those with brain metastases. In the event of hemorrhage from brain metastases, selective arterial cannulation and embolization may be preferred to avoid incomplete surgery and a range of postoperative complications that may arise from emergency open surgery. After treatment, the social, emotional, cognitive, and spiritual functions of the two groups increased significantly. The results fully confirm that chemotherapy treatment for patients with malignant trophoblastic tumors brain metastatic can improve the quality life of patients can feel the warmth of family, and better return to society, which is of great significance to the improvement of patients' quality of life.

## 7. Conclusions

The present study excluded the influence of confounding factors such as primary and metastatic foci on the results. Although PFS and OS were significantly longer in this study compared to other studies, because it was a single-centre, prospective, single-arm study, future multicentre, prospective, randomised controlled clinical studies are needed to understand the effect of treatment of brain metastases from zygotic tumours and the prognostic risk factors during pregnancy.

## Figures and Tables

**Figure 1:** Analysis of the treatment effects.

**Figure 2:** PFS graph for the whole group.

**Figure 3:** OS curves for the whole group.

**Figure 4:** Analysis of toxicity and adverse reactions.

**Figure 5:** Quality of life analysis at different time points after treatment.

**Table 1:** Univariate analysis of the effect of OS and PFS on patients ($\bar{x}\pm s$).

Factor	Median OS (month)	*P* value	Median PFS (month)	*P* value
Gender		0.026		0.035
Male	21		17.5	
Female	10.5		11.6	

Number of metastases		0.01		0.083
>3	13		11.3	
=3	25		21	

RPA classification		0		0.125
Level 1	25		21	
Level 2	11		11.7	

MMSE score before radiotherapy		0.09		0
27–30 points	20		21	
<27 points	10.3		9.5	

Extracranial metastasis				0.012
Have			11.6	
Nothing			21	

**Table 2:** Multifactor analysis affecting patients' OS and PFS.

Factor	Regression coefficient	*x* ^2^ value	*P* value	RR value	95% CI
RPA rating (OS)	−2.019	9.487	0.002	0.133	0.037–0.48
MMSE score (PFS) before radiotherapy	−2.337	11.019	0.01	0.097	0.024–0.384

**Table 3:** Toxic adverse effects in patients receiving TMZ combined with whole-brain radiotherapy (cases).

Toxic adverse reaction	Classification of toxic and adverse reactions				
	0	1	2	3	4
Hematological toxicity					
Leucopenia	10	10	6	5	0
Thrombocytopenia	10	4	10	7	0
Both decreased	19	8	2	2	0

Gastrointestinal toxicity					
Nausea and vomiting	5	10	10	6	0
Diarrhea	19	10	2	0	0

## Data Availability

The data used to support the findings of this study are available from the corresponding author upon request.
